The article "Ultrasound Assessment of the Relevance of Liver, Spleen, and Kidney Dimensions with Body Parameters in Adolescents" was published in 2022. Journal: Comput Math Methods Med.

# Ultrasound Assessment of the Relevance of Liver, Spleen, and Kidney Dimensions with Body Parameters in Adolescents

**DOI:** 10.1155/2022/9150803

**Published:** 2022-07-04

**Authors:** Ying Huang, Yumei Zheng, Cuncheng Zhang, Shigen Zhong

**Affiliations:** ^1^Department of Ultrasound, Chongqing General Hospital, Chongqing 401147, China; ^2^Department of Ultrasound, Hangzhou Hospital of Zhejiang Medical and Health Group, Hangzhou 310022, China; ^3^Department of Health Management Center, Chongqing General Hospital, Chongqing 401147, China

## Abstract

**Objective:**

Ultrasound is a practical imaging modality for screening and identification of anomalies in the organs. This study used ultrasonography to examine the association between body parameters and dimensions of the normal liver, spleen, and kidney in adolescents based on ultrasound examination results.

**Methods:**

A total of 300 junior and senior high school teenagers receiving routine health check-ups in our hospital from January 2020 to January 2021 were included. Their height and weight were measured, and their body surface area (BSA) and body mass index (BMI) were calculated. Ultrasound imaging was employed to obtain information such as the length and volume of the liver, gallbladder, spleen, and kidney. Besides, the correlation of body parameters such as gender, age, height, weight, BSA, and BMI with visceral dimension was investigated using the Pearson test and multiple regression analysis, respectively.

**Results:**

We observed that the abdominal organs of adolescents were enlarged with age. The span and volume of the liver and the length and volume of the right kidney were significantly larger in boys than in girls. The age, BSA, and BMI were positively correlated with the liver span and spleen length, as well as the left and right kidney lengths. Additionally, age, BSA, and BMI were identified as important predictors for dimensions of the spleen, liver, and kidney.

**Conclusions:**

Body parameters are notably associated with the dimensions of the liver, spleen, and kidney and could be utilized as predicting factors for the liver, spleen, and kidney dimensions.

## 1. Introduction

As the largest peripheral immune organ, the spleen is the settlement site for T and B cells and has a direct link with immune function [1]. Antigenic stimulus to the body can induce lymphoid tissue proliferation and result in the proliferation and immune response of lymphocytes, plasma cells, and macrophages, which can cause the occurrence of antibodies and a large number of T effector cells, thereby inducing splenomegaly [2]. Macrophage is abundant in the liver. Antigenic stimuli can induce macrophage proliferation and contributes to hepatomegaly [3]. In addition, hepatosplenomegaly can be caused by some metabolic substance deposition or abnormal cell infiltration, posthepatitic cirrhosis, chronic hepatitis, and various hematological diseases like acute leukemia, chronic leukemia, thalassemia, myelodysplastic syndrome, hemophagocytic syndrome, hemolytic anemia, etc. [4]. Moreover, hepatosplenomegaly can sometimes be the initial symptoms of some diseases. The basic functions of the kidney include urine production, excretion of metabolites, maintenance of fluid and acid-base balance, and endocrine function [5]. Kidneys can be enlarged when patients suffer from diabetic nephropathy, hydronephrosis, polycystic kidney disease, and acute glomerulonephritis [6]. As many factors are associated with hepatosplenomegaly and renomegaly, it is difficult to clinically diagnose them without a clear medical history.

Clinical assessment of the liver is accomplished by palpating the extension degree of the liver below the costal margin and the span of dull percussion note [7]. Normal liver margin can be observed 2 cm below the right costal margin, while neonates can be observed 3.5 cm below the costal margin in the midclavicular line [8]. The spleen is palpable when it reaches at least twice or thrice its normal size, although it may be palpable in 10% of healthy children and 15% of newborns [9]. Palpation and percussion have been proven to be relatively inaccurate in measuring spleen and liver dimensions [8, 10]. The kidney size cannot be measured by routine health check-ups, and the enlarged kidney can only be palpated when it develops to a certain degree [11]. At present, hepatomegaly, splenomegaly, and renomegaly are mainly detected with physical examination, abdominal ultrasound, abdominal X-ray, computed tomography (CT), and magnetic resonance imaging (MRI). However, aside from the disadvantage of radiation and high cost, abdominal X-ray, routine CT, and MRI cannot detect the hemodynamic changes of these organs. To identify the cause of splenomegaly, bone marrow puncture is the gold standard for splenomegaly caused by hematological diseases [12]. Liver biopsy is the most acknowledged method for diagnosing splenomegaly caused by liver diseases [13]. However, both of the above methods are invasive. Ultrasonography, as a practical, readily available, cheap, noninvasive, and clinically satisfactory accuracy, especially for routine examination purposes, is commonly used to assess the size of abdominal organs. But due to the lack of standard measurement data for the accurate dimensions of the liver, spleen, and kidneys in adolescents, either for screening or routine health check-up purposes, interpreting ultrasonography results could be difficult in clinical practice and might sometimes lead to misdiagnosis or missed diagnosis, especially in young adolescents and for small potential lesions or asymptomatic anomalies that could affect the dimensions of their liver, spleen, and kidneys but are not evident unless the ultrasound is meticulously performed and the measurements are analyzed. Thus, it is important to have a referential range for the dimensions of the liver, spleen, and kidneys as it could potentially help to identify potential anomalies.

Therefore, this study used ultrasonography to assess the dimensions of the liver, spleen, and kidney in healthy adolescents, and based on the assessment results, the correlation of the liver, spleen, and kidney dimensions with body parameters was analyzed. The objectives of this study were to provide data supporting the clinical assessment of potential pathological conditions in the liver, spleen, and kidney of adolescents.

## 2. Materials and Methods

### 2.1. Study Subjects

The data of a total of 300 junior and senior high school adolescents who underwent routine health check-ups in our hospital from January 2020 to January 2021 were collected. Inclusion criteria as follows: (1) adolescents aged 13 to17 years old [14]; (2) provided detailed clinical history; (3) had no infection or solid lesion in their liver, kidney, and spleen; and (4) volunteered to engage in the investigation, and the guardian's informed consents were acquired. Exclusion criteria are as follows: (1) adolescents who suffered from any infectious, inflammatory, hematological, malignant, congestive, or collagen diseases that affected the size of the liver, kidney, or spleen; (2) diagnosed with acute or chronic hepatitis, jaundice, or chronic renal failure; (3) had fever, lymphadenopathy, macular or maculopapular rash within the past three months; and (4) suffered from dwarfism, gigantism, malnutrition, or obesity. Exclusion criteria of imaging are as follows: adolescents were found with (1) abnormal location, shape, and echo structure of the liver, kidney, and spleen; (2) solid mass lesions; and (3) cysts of the liver, kidney, and spleen, accessory spleen, or hydronephrosis. The general information of the subjects was recorded, and all subjects signed the informed consent form. This study was approved by the Ethics Committee of Chongqing General Hospital (KYS2022-014-01).

### 2.2. Detection of Human Body Parameters

The height of all subjects was measured (accuracy: 0.1 cm) using a domestic cylindrical height measurement corrected by a professional before use. During the measurement, the subjects were barefoot and upright on the central position of the plate table. The average of two consecutive measurements would be taken as the final value of height, with a difference between the two measurements less than 0.5 cm. The subjects' body weight was measured using an electronic weight scale per national standards (accuracy: 0.1 kg). During measurements, subjects were required to wear light clothes and stand on the central position of the table. Body weight was read after the scale reading was stable. Light clothing was defined as casual shirts, shorts, or trousers. If the patients wore jackets or comparatively thicker clothing, they were advised to remove them for the experiment's purposes.

After the height and weight measurements, body surface area (BSA) and body mass index (BMI) were calculated as the following formula: BSA = ([Height (cm) × Weight (kg)]/3600) ½, BMI = Weight (kg)/[Height (cm)].

### 2.3. Ultrasound

Subjects lay on their back to obtain an optimal view of the liver and gallbladder. Longitudinal views were taken using a B-mode ultrasound machine (Philips IU22) at the midclavicular midline positions to measure the span and volume of the liver. The anteroposterior diameter (AP diameter) was also measured at the midpoint of the longitudinal diameter. Longitudinal and transverse measurements of the gallbladder were performed by subcostal or intercostal approaches during deep inspiration in the supine position, and the contents were assessed (clear echoes, cholestasis). For spleen measurements, lateral decubitus position was required, with longitudinal dimension measured between the uppermost medial point and the lowermost lateral point of the spleen. The spleen length and volume were recorded. Renal measurements were performed in the lateral decubitus position, and the length of the kidney was obtained by measuring the bipolar length of the kidney. Besides, the AP diameter of the kidney was measured, and the length and volume of the left and right kidneys were recorded. Organ volume was calculated using the following formula: volume = length × width × AP diameter × 0.52.

### 2.4. Statistical Analysis

SPSS 24.0 was used for the data analysis; one-way analysis of variance for comparison between multiple groups; while independent samples *t*-test for comparison between two groups; Pearson test for analysis of the correlation between body parameters and abdominal organ size; and multivariate regression for the analysis of the predictive effect of body parameters on abdominal organ size. Differences were considered statistically significant when *P* < 0.05.

## 3. Results

### 3.1. General Information of Subjects

In total, 150 boys and 150 girls were involved in this study (age range, 13-17 years). We observed that their height, weight, BMI, and BSA were increased with age for both the girls and boys (Table 1).

### 3.2. Abdominal Organ Size Results in Adolescents of Different Ages

The subjects' liver span, gallbladder echoes, and contents, as well as the length of spleen and kidney, were measured using ultrasound (Figures 1(a)–1(f)), and the size of each organ was divided according to age and gender. The results revealed that the liver span and the length of the left and right kidneys were increased with age in all subjects. However, spleen length showed a decreased tendency in boys at 15 years old and an increased tendency at 16 and 17 years old. For girls, their liver span and spleen length tended to decrease at the age of 16, while they increased again at the age of 17. Besides, the cases of subjects with cholestasis increased when they were 16 and 17 years old. In addition, boys had significantly higher liver span, liver volume, right kidney length, and right kidney volume than girls, while there were no significant differences in spleen length and volume and left kidney length and volume (Table 2).

### 3.3. Relevance between Abdominal Organ Dimensions and Body Parameters

The Pearson test was adopted to analyze the correlation of age, BSA, and BMI with abdominal organ size in all subjects, and the results were plotted as a heat map. According to the results, the subjects' age, BSA, and BMI were positively correlated with the liver span, spleen length, and left and right kidney length in both boys and girls (Figure 2).

### 3.4. Multivariate Regression Analysis for the Relationship between Abdominal Organ Size and Body Parameters

Multiple regression analysis was performed to analyze the correlation of abdominal organ size with age, BMI, and BSA of the study subjects. The results showed that, regardless of gender, age served as an important predictor for spleen length; BSA as a predictor for liver span and left and right kidney length; and BMI for liver span, spleen length, and right kidney length. Upon further analysis, age was identified as an important predictor for the liver span in boys; BSA as a crucial predictor for the liver span, spleen length, and left and right kidney length; and BMI for the right kidney length, whereas for girls, age acted as a significant predictor of liver span and spleen length; BSA as a significant predictor of the liver span and left kidney length; and BMI as a predictor of the length of spleen and the kidneys (Table 3).

## 4. Discussion

As an important clinical imaging tool, ultrasound can assist in diagnosing various diseases with the advantages of being invasive, safe, yield rapid results, and much cheaper than CT and MRI [15]. Timely detection of the abnormal size of these organs can contribute to early diagnosis and treatment since various disease states can affect the dimension of the liver, spleen, and kidneys. Some previous studies have reported the range of normal ultrasound parameters of abdominal organs in infants and children [16–18], but the range for adolescents has not been presented in China. Unlike the normal range of organ size in adults, the organ size of minors was related to their growth and development. Therefore, the normal value of liver, spleen, and kidney size measured by ultrasound varies with the age of minors [19, 20]. In this study, we discovered that liver span and the length of spleen and kidney in adolescents increased with age, which is consistent with preceding studies.

However, the study results on the size of abdominal organs showed some differences due to gender. Some studies indicated that, regardless of the groups of infants [21] or children [19], no statistical significance could be spotted in the size of the liver, spleen, and kidney in different genders. But some researchers have presented that there might be differences in the organ size between genders. For example, Akinlade et al. [22], in a study of 1,000 pupils in southwest Nigeria, reported that liver span and spleen length were significantly larger in boys than in girls, while the location of the left lobe of the liver was higher in girls; but there was no significant difference in the size of the kidneys between boys and girls. In this study, there were differences in some abdominal organ dimensions between subjects of different genders. For instance, boys had higher values than girls in the span and volume of liver and right kidney, which may be explained by physical differences between males and females. However, the length and volume of the spleen and left kidney displayed no variance.

Previous studies have stated that the longitudinal lengths of the liver, spleen, and kidney correlate most with body parameters [19, 23]. Our study was concordant with these findings. Overall, in this study, the subjects' age, BSA, and BMI were positively correlated with the liver span, the length of the spleen, and the length of the left and right kidneys. Multivariate regression analysis revealed the following: firstly, age could be used as an important predictor of spleen length. Secondly, BSA could predict liver span and the length of the left and right kidneys; lastly, BMI could serve as a critical predictor of liver span, spleen length, and right kidney length.

However, the small sample size of this study may have affected the study findings. Further, our results might not be enough to quantify the relevance between body parameters and abdominal organ dimension. A larger sample size and multicenter setting could provide more evidence and feasible data for accurate clinical estimation of abdominal organ size in adolescents.

## 5. Conclusion

In summary, this study is the first report to analyze the relationship between body parameters and abdominal organ size in China. Besides, we found a significant relevance between body parameters such as age, BSA, and BMI with the dimensions of the liver, spleen, and kidney, suggesting that body parameters could act as predictors for abdominal organ size but could vary gender differences.

## Figures and Tables

**Figure 1:** Ultrasound findings of the liver, gallbladder, spleen, and kidney of one subject. (a–f) Ultrasound examination for liver span (a), clear echoes (b), and cholestasis (c) in the gallbladder, spleen length (d), left kidney length (e), and right kidney length (f).

**Figure 2:** Relevance between organ size and body parameters.

**Table 1:** General information of subjects.

Gender	Age	Height (cm)	Weight (cm)	BMI (kg/m^2^)	BSA(m^2^)
Male (*n* = 150)	13	145.43 ± 4.46	36.18 ± 3.61	17.06 ± 0.76	1.21 ± 0.08
	14	149.57 ± 4.75	40.18 ± 3.62	17.92 ± 0.63	1.29 ± 0.08
	15	153.77 ± 5.04	44.18 ± 3.61	18.65 ± 0.52	1.37 ± 0.08
	16	158.00 ± 4.72	48.25 ± 3.78	19.29 ± 0.48	1.45 ± 0.08
	17	162.43 ± 5.08	53.00 ± 4.28	20.06 ± 0.43	1.55 ± 0.09
Female (*n* = 150)	13	140.10 ± 4.33	36.78 ± 2.83	18.71 ± 0.44	1.20 ± 0.06
	14	143.97 ± 4.24	40.78 ± 2.83	19.65 ± 0.38	1.28 ± 0.06
	15	148.20 ± 4.21	43.78 ± 2.84	19.91 ± 0.37	1.34 ± 0.06
	16	152.03 ± 4.13	46.28 ± 2.83	20.00 ± 0.31	1.39 ± 0.06
	17	155.57 ± 4.98	49.45 ± 3.08	20.41 ± 0.26	1.47 ± 0.07

**Table 2:** Dimensions of abdominal organs in subjects of different ages.

Gender	Age (year)	Liver span (cm)	Liver volume (cm^3^)	Spleen length (cm)	Spleen volume (cm^3^)	Left kidney length (cm)	Left kidney volume (cm^3^)	Right kidney length (cm)	Right kidney volume (cm^3^)	Gallbladder contents
Male	13	12.14 ± 0.45	465.11 ± 12.94	5.17 ± 0.10	31.01 ± 4.29	10.77 ± 0.08	82.92 ± 2.72	9.15 ± 0.08	80.30 ± 8.13	4
	14	12.60 ± 0.45	494.96 ± 14.32	5.57 ± 0.10	37.56 ± 2.41	10.93 ± 0.16	91.18 ± 2.73	9.42 ± 0.14	83.62 ± 5.13	4
	15	13.27 ± 0.49	522.40 ± 19.10	5.37 ± 0.10	43.83 ± 2.41	11.13 ± 0.18	97.44 ± 2.81	9.67 ± 0.26	94.20 ± 3.06	5
	16	14.02 ± 0.62	550.43 ± 25.28	5.87 ± 0.10	50.17 ± 2.35	11.31 ± 0.24	107.04 ± 2.99	9.96 ± 0.32	100.22 ± 2.51	11
	17	14.89 ± 0.79	578.43 ± 32.08	6.57 ± 0.10	60.44 ± 2.35	11.49 ± 0.29	117.75 ± 3.06	10.27 ± 0.34	110.22 ± 4.41	15
Female	13	12.20 ± 0.53	451.08 ± 15.85	5.15 ± 0.11	32.30 ± 5.26	10.74 ± 0.13	84.83 ± 2.49	9.00 ± 0.10	78.65 ± 4.71	5
	14	12.70 ± 0.50	481.99 ± 28.77	5.49 ± 0.13	39.55 ± 6.40	10.92 ± 0.16	92.00 ± 2.10	9.24 ± 0.10	83.64 ± 5.01	6
	15	13.17 ± 0.51	506.35 ± 23.31	5.87 ± 0.19	44.45 ± 4.23	11.00 ± 0.30	99.16 ± 8.53	9.49 ± 0.13	87.93 ± 4.05	5
	16	12.82 ± 0.51	530.34 ± 18.63	5.66 ± 0.17	51.37 ± 3.14	11.23 ± 0.30	106.32 ± 10.26	9.69 ± 0.23	92.21 ± 3.21	11
	17	13.20 ± 0.54	555.03 ± 15.42	6.00 ± 0.26	58.43 ± 2.37	11.45 ± 0.27	113.48 ± 5.26	9.94 ± 0.26	96.44 ± 2.62	16

**Table 3:** Relationship between abdominal organ size and body parameters predicted by multivariate regression analysis.

Parameters	Total		Male		Female	
	Standardized regression coefficient	*P*	Standardized regression coefficient	*P*	Standardized regression coefficient	*P*
Liver span						
Age	0.036	0.119	0.389	≤0.001	0.769	≤0.001
BMI	0.521	≤0.001	-0.132	0.163	0.012	0.546
BSA	0.981	≤0.001	0.706	≤0.001	0.404	≤0.001
Spleen length						
Age	0.123	≤0.001	-0.019	0.712	0.254	0.005
BMI	0.459	≤0.001	-0.048	0.668	0.188	0.030
BSA	0.056	0.194	0.380	≤0.001	0.028	0.412
Left kidney length						
Age	-0.082	0.117	-0.020	0.709	-0.102	0.156
BMI	0.458	≤0.001	-0.013	0.748	0.241	0.019
BSA	0.424	≤0.001	0.460	≤0.001	0.473	≤0.001
Right kidney length						
Age	0.051	0.105	-0.111	0.392	-0.045	0.501
BMI	0.013	0.356	0.298	≤0.001	0.335	≤0.001
BSA	0.512	≤0.001	0.699	0.009	-0.098	0.398

## Data Availability

The data used to support the findings of this study are available from the corresponding author upon request.
